# Overexpression of lncRNA ANRIL up-regulates VEGF expression and promotes angiogenesis of diabetes mellitus combined with cerebral infarction by activating NF-κB signaling pathway in a rat model

**DOI:** 10.18632/oncotarget.14468

**Published:** 2016-12-04

**Authors:** Bo Zhang, Dan Wang, Tie-Feng Ji, Lei Shi, Jin-Lu Yu

**Affiliations:** ^1^ Department of Neurosurgery, The First Hospital of Jilin University, Changchun, P.R. China; ^2^ Department of Ophthalmology, The First Hospital of Jilin University, Changchun, P.R. China; ^3^ Department of Radiology, The First Hospital of Jilin University, Changchun, P.R. China

**Keywords:** LncRNA ANRIL, diabetes mellitus, cerebral infarction, NF-κB signaling pathway, vascular endothelial growth factor

## Abstract

**Objective:**

This study aimed to explore the effects of lncRNA ANRIL on vascular endothelial growth factor (VEGF) and angiogenesis in diabetes mellitus (DM) combined with cerebral infarction (CI) through NF-κB signaling pathway.

**Methods:**

Adult male Wistar rats were randomly divided into control group and DM + CI group, and the DM + CI group were subdivided into Vector, shANRIL, PDTC, pcDNA-ANRIL, and pcDNA-ANRIL + PDTC groups. VEGF and FMS-like tyrosine kinase (FLT-1) expressions were measured by immunohistochemistry and endothelium dependent microvessel density (MVD) was detected by differentiation 31 (CD31) and para-amiuosalicylic acid (PAS) double staining. The qRT-PCR was applied to measure mRNA expressions of VEGF, FLT-1, Kinase insert domain protein receptor (FLK-1) and NF-κB, and Western blotting was conducted to detected expressions of VEGF, NF-κB and p-I?B/I?B.

**Results:**

Compared with the control group, protein expressions of VEGF, NF-κB, p-I?B/I?B, expression of ANRIL, and mRNA expressions of VEGF, FLT-1 and NF-κB were increased in the DM + CI group. Compared with the Vector group, protein expressions of VEGF, NF-κB, p-I?B/I?B, expression of ANRIL, mRNA expressions of VEGF, FLT-1 and NF-κB, and endothelium dependent MVD were increased in the pcDNA-ANRIL group, while decreased in the shANRIL group and PDTC group. Compared with the pcDNA-ANRIL group, protein expressions of VEGF, NF-κB, p-I?B/I?B, expression of ANRIL, mRNA expressions of VEGF, FLT-1 and NF-κB, and endothelium dependent MVD were decreased in the pcDNA-ANRIL + PDTC group.

**Conclusion:**

Overexpressed lncRNA ANRIL upregulates VEGF and promotes angiogenesis by activating NF-κB signaling pathway in DM + CI rats.

## INTRODUCTION

Diabetes mellitus (DM) is characterized by complicated metabolic disorders and has been considered as an common chronic disease in the world, with an incidence approximate to 382 million in 2013, which is classified to be two types including type 1 DM (T1DM) and type 2 DM (T2DM) [1]. It’s found that DM played an independent role of increasing the risk of cerebral infarction (CI) [2], where CI might be induced by serious metabolic dysfunction [3]. The common initial manifestation of CI might be caused by arterial occlusion, and there is a high mortality of patients when CI combined with T2DM, where the major pathology of CI is thrombosis [4]. CI was not only stated to be developed with DM by its hypercoagulable state but also a complication of diabetic ketoacidosis in plenty of children all over the world [5]. CI leads to cell membrane depolarization and activating glutamate receptors, and at same time, the death or survival signals of cells were transformed [6]. The early diagnosis and prompt treatment of CI are supposed to be explored as early as possible, especially multiple metabolic pathways, because the uncertain diagnosis causes the poor administration of plasminogen activator in the present state [7]. Thus finding more molecular levels related to DM complicated with CI would be beneficial for better clinic treatment.

Long non-coding RNA (lncRNA), identified as non-protein-coding RNAs which have long length with over 200 nucleotides, involves in many biological actions including cell growth and proliferation and so on [8]. Antisense non-coding RNA in the INK4 locus (ANRIL), belonging to the lncRNA family, widely exits in various human cancers, and also is regarded as a dangerous existence in breast cancer, gliomas and other several cancers proved by increasing studies [9]. ANRIL is a 3.8 kb lncRNA, reversing from a gene cluster named INK4B-ARF-INK4A in the direction, besides, ANRIL knockdown was found that can inhibit proliferation either *in vivo* or vitro [10]. A previous study demonstrated that ANRIL influences nuclear factor-κB (NF-κB) pathway in which increased ANRIL might regulate the NF-κB expressions [11]. ANRIL is supposed to be essential in mediating Chr9p21 associations and for treating a number of human diseases as a target molecule, in particular, regulating ANRIL expressions was found to be related to risk variants of DM [12]. Therefore, this study aims to find whether ANRIL has an influence on DM complicated with CI, and further discuss the mechanism of ANRIL in DM complicated with CI patients. This study supposes that ANRIL regulates NF-κB signal pathway to change the expressions of vascular endothelial growth factor (VEGF) and angiogenesis in DM + CI rats.

## RESULTS

### Successful establishment of rat models

Fifty-six rats received alloxan injection through abdomen, after which, whose fasting blood glucose was above 16.7 mmol/L. Within the next 1 month, 5 rats died and fasting blood glucose of the rest 51 ones was above 16.7 mmol/L, which making model success rate at 91.07%. After successful DM models were established, rats showed remarkable weight loss, increased water intake, food intake and urinary production, filthy and dark furs as well as frequently fluctuated blood sugar at relatively high level. Based on successful DM models, CI models were established, during which process 5 rats died and the rest 46 ones survived. And neurological function change of various degrees appeared in rats models whose NSS were remarkably higher than healthy control group (*P* < 0.05), which could be seen from Table 2. All together 46 rats model with DM complicated with CI were successfully established, which making success rate standing at 82.14%. In each group, 8 rats were selected at random for TTC staining, in which normal tissues were in red and ischemic infarct area in pale white. CI volume was detected to be (21.26 ± 3.15) %, staining result of which was revealed in Figure 1.

**Figure 1:** Comparison of ischemic infarct area between the control group and DM + CI group by TTC staining (A, Ischemic infarct area in the control group; B, Ischemic infarct area in the DM + CI group. Normal tissues were in red and ischemic infarct areas were in pale white. Compared with the control group, the DM + CI group had more ischemic infarct area)Notes: TTC, triphenylte-trazolium chloride; DM, diabetes mellitus; CI, cerebral infarction.

**Figure 2:** Comparison of pathological changes between the control and DM + CI groups by HE staining (**A**, Pathological changes in the control group; **B**, Pathological changes in the DM + CI group; **C**, Histogram of neuronal cell number in the control group and DM + CI group. Gap between neural neural cells in CI was widened area and neuron numbers were decreased in the center; data were showed in mean ± standard deviation). Notes: HE, haematoxilin-eosin; DM, diabetes mellitus; CI, cerebral infarction; *, compared with the control group, *P* < 0.05.

**Table 1:** The amplified primer sequences

Primers	Primer sequences (5′ - 3′)
VEGF upstream	GCTCTCTTGGGTGCACTGGA
VEGF downstream	CACCGCCTTGGCTTGTCACA
FLT-1 upstream	TCATGCAAGCGGGCCAGACTCTCTTTC
FLT-1 downstream	ATCTCACGGGGCTCGGCGGGCTTATTT
FLK-1 upstream	CATTGTGTCCTGCATCCGGGATAACCT
FLK-1 downstream	TGTACACGATGCCATGCTCGTCACTGA
NF-κB upstream	AACACTGCCGACCTCAAGAT
NF-κB downstream	CATCGGCTTGAGAAAAGGAG
ANRIL upstream	TTATGCTTTGCAGCACACTGG
ANRIL downstream	GTTCTGCCACAGCTTTGATCT
GAPDH upstream	ACAGCAACAGGGTGGTGGAC
GAPDH downstream	TTTGAGGGTGCAGCGAACTT

Notes: VEGF, vascular endothelial growth factor; FLT-1, FMS-like tyrosine kinase; FLK-1, Kinase insert domain protein receptor; NF-κB, nuclear factor-κB; ANRIL, antisense non-coding RNA in the INK4 locus; GAPDH, glyceraldehyde phosphate dehydrogenase.

**Table 2:** Neurological severity scores (NSS) of the control group and DM + CI group

Groups	n	Scores	P
Control group	6	0	
DM + CI group	6	3.20 ± 1.03	< 0.001

Notes: DM, diabetes mellitus; CI, cerebral infarction.

Comparison of pathological changes between the control and DM + CI groupsObservation under light microscope found that DM + CI group saw widened gap between neural cells in CI area, decreased neuron numbers in the center, obvious hemorrhagic change and such symptoms of cell necrosis as karyopyknosis in remaining neurons and tissue looseness, which can be seen from

### Comparisons of VEGF, NF-κB and p-IκB/ IκB protein expressions in each group

As shown in Figure 3A, compared to rats in control group, those in DM + CI group saw a more remarkable increase in protein expressions of VEGF, NF-κB and p-IκB/IκB in brain tissues (both *P* < 0.05). Further efforts were made to detect NF-κB signaling pathway and VEGF protein expression in brain tissues with over-expressed or knocked lncRNA ANRIL so as to verify the effect of lncRNA ANRIL on rat model with DM complicated with CI. It was revealed in Figure 3B that over-expression of lncRNA ANRIL resulted in a more notable increase in protein expression levels of VEGF, NF-κB and p-IκB/IκB than Vector group (all *P* < 0.05), while knockout of lncRNA ANRIL brought about a more obvious decrease in protein expression levels of VEGF, NF-κB and p-IκB/IκB than Vector group (all *P* < 0.05). After using inhibitor PDTC to inhibit NF-κB signaling pathway, protein expression levels of VEGF, NF-κB and p-IκB/IκB were more remarkably reduced than Vector group, and protein expression levels of VEGF, NF-κB and p-IκB/IκB were reduced after injected inhibitor PDTC of over-expressed lncRNA ANRIL than over-expression of lncRNA ANRIL (all *P* < 0.05).

**Figure 3:** Comparisons of VEGF, NF-κB and p-IκB/IκB protein expressions in each group by Western blotting (**A**, Comparisons of VEGF, NF-κB and p-IκB/IκB Protein expression in the control group and DM + CI group; **B**, Comparisons of VEGF, NF-κB and p-IκB/IκB Protein expression in DM + CI groups. Compared with the Vector group, protein expression of VEGF, NF-κB and p-IκB/IκB were increased in the pcDNA-ANRIL group, while protein expression of VEGF, NF-κB and p-IκB/IκB were decreased in the shANRIL group and the PDTC group. Compared with the pcDNA-ANRIL group, protein expression of VEGF, NF-κB and p-IκB/IκB were decreased in the pcDNA-ANRIL + PDTC group; Relative expression of protein were showed in column chart, data were showed in mean ± standard deviation). Notes: VEGF, vascular endothelial growth factor; NF-κB, nuclear factor-κB; The Vector group, injected with 800 ng/kg empty plasmid; The shANRIL group, injected with 800 ng/kg lncRNA ANRIL knockout plasmid; The PDTC group, injected with 800 ng/kg NF-κB inhibitor pyrrolidine dithiocarbamate (PDTC); The pcDNA-ANRIL + PDTC group, injected with PDTC after lncRNA ANRIL overexpression; DM, diabetes mellitus; CI, cerebral infarction; *, compared with the control/ Vector group, *P* < 0.05.

### Comparisons of ANRIL expression and VEGF, FLT-1, FLK-1 and NF-κB mRNA expressions in each group

As was revealed in Figure 4A, qRT-PCR was employed to detect ANRIL, VEGF, FLT-1, FLK-1 and NF-κB mRNA expression levels in rats’ tissues in control group and DM + CI group, showing that DM + CI group had a more apparent increase in ANRIL expression level than control group (*P* < 0.05) and more remarkably upregulated VEGF, FLT-1 and NF-κB expressions than control group (all *P* < 0.05), while no statistical difference was shown in FLK-1 mRNA expression between the two groups (*P* > 0.05). It was shown in Figure 4B that transfection efficiency detection of over-expressed ANRIL found that ANRIL expression increased by 0.88-fold while knockout of ANRIL made ANRIL expression decrease by 40%. DM + CI rat model with over-expressed lncRNA ANRIL showed more obviously upregulated VEGF, FLT-1 and NF-κB mRNA expressions than Vector group (all *P* < 0.05). However, when lncRNA ANRIL was knocked and receiving PDTC treatment, the VEGF, FLT-1 and NF-κB mRNA expressions were more apparently downregulated than Vector group (all *P* < 0.05), while FLK-1 mRNA expression demonstrated no difference before and after treatment (*P* > 0.05). Inhibitor PDTC was injected after lncRNA ANRIL overexpression, the VEGF, FLT-1 and NF-κB mRNA expressions were significantly decreased than over-expressed lncRNA ANRIL (all *P* < 0.05), while FLK-1 mRNA expression demonstrated no difference before and after treatment (*P* > 0.05).

**Figure 4:** Comparisons of ANRIL expression and VEGF, FLT-1, FLK-1 and NF-κB mRNA expressions in each group by qRT-PCR (**A**, Comparisons of ANRIL expression and VEGF, FLT-1, FLK-1 and NF-κB mRNA expressions in the control group and DM + CI group; **B**, Comparisons of ANRIL expression and VEGF, FLT-1, FLK-1 and NF-κB mRNA expressions in DM + CI groups. Expression of lncRNA ANRIL was increased after transfected with over-expressed lncRNA ANRIL, while expression of lncRNA ANRIL was decreased after transfected with inhibitor lncRNA ANRIL. Compared with the Vector group, expression of VEGF, FLT-1, FLK-1 and NF-κB mRNA were increased in the pcDNA-ANRIL group, whereas expression of VEGF, FLT-1, FLK-1 and NF-κB mRNA were decreased in the shANRIL group and the PDTC group. Compared with the pcDNA-ANRIL group, expression of VEGF, FLT-1, FLK-1 and NF-κB mRNA were decreased in the pcDNA-ANRIL + PDTC group). Notes: qRT-PCR, quantitative real-time polymerase chain reaction; FLT-1, FMS-like tyrosine kinase; FLK-1, kinase insert domain protein receptor; NF-κB, nuclear factor-κB; PDTC, pyrrolidinedithiocarbamic acid; VEGF, vascular endothelial growth factor; lncRNA, long non-coding RNA; The Vector group, injected with 800 ng/kg empty plasmid; The shANRIL group, injected with 800 ng/kg lncRNA ANRIL knockout plasmid; The PDTC group, injected with 800 ng/kg NF-κB inhibitor pyrrolidine dithiocarbamate (PDTC); The pcDNA-ANRIL + PDTC group, injected with PDTC after lncRNA ANRIL overexpression; DM, diabetes mellitus; CI, cerebral infarction; *, compared with the Vector group, *P* < 0.05.

### Comparisons of VEGF and FLT-1 expressions in each group

According to immunohistochemical results, Figure 5 showed visible VEGF positively stained vessels near the infarct focus in cytoplasm in brownish yellow, but no VEGF protein expression was detected in ischemic center and non-ischemic regions. Compared to Vector group, over-expressed lncRNA ANRIL led to an increase in VEGF expression; however, knockout of lncRNA ANRIL and injection of PDTC brought about a decrease in VEGF expression. Compare to over-expressed lncRNA ANRIL, injection of inhibitor PDTC after lncRNA ANRIL overexpression showed an increased expression of VEGF. Positive staining of FLT-1 was in brownish yellow. Compared to Vector group, over-expressed lncRNA ANRIL resulted in an increased expression of FLT-1 while its knockout and PDTC injection incurred a reduced FLT-1 expression. Compare to over-expressed lncRNA ANRIL, injection of inhibitor PDTC after lncRNA ANRIL overexpression showed a reduced expression of FLT-1 (Figure 6).

**Figure 5:** Comparisons of VEGF expressions in each group by IHC (× 400) (**A**, VEGF expressions in the Vector group; **B**, VEGF expressions in the pcDNA-ANRIL group; **C**, VEGF expressions in the shANRIL group; **D**, VEGF expressions in the PDTC group; **E**, VEGF expressions in the pcDNA-ANRIL + PDTC group. Compared with the Vector group, expression of VEGF was increased in the pcDNA-ANRIL group, while expression of VEGF was decreased in the shANRIL group and the PDTC group. Compared with the pcDNA-ANRIL group, expression of VEGF was evaluated in the pcDNA-ANRIL + PDTC group). Notes: IHC, immunochemistry; PDTC, pyrrolidinedithiocarbamic acid; VEGF, vascular endothelial growth factor; ANRIL, antisense non-coding RNA in the INK4 locus; The Vector group, injected with 800 ng/kg empty plasmid; The shANRIL group, injected with 800 ng/kg lncRNA ANRIL knockout plasmid; The PDTC group, injected with 800 ng/kg NF-κB inhibitor pyrrolidine dithiocarbamate (PDTC); The pcDNA-ANRIL + PDTC group, injected with PDTC after lncRNA ANRIL overexpression; DM, diabetes mellitus; CI, cerebral infarction.

**Figure 6:** Comparisons of FLT-1 expressions in each group by IHC (× 400) (**A**, FLT-1 expressions in the Vector group; **B**, FLT-1 expressions in the Vector group in the pcDNA-ANRIL group; **C**, FLT-1 expressions in the shANRIL group; **D**, FLT-1 expressions in the PDTC group; **E**, FLT-1 expressions in the pcDNA-ANRIL + PDTC group. Compared with the Vector group, expression of FLT-1 was increased in the pcDNA-ANRIL group, while expression of FLT-1 was decreased in the shANRIL group and the PDTC group. Compared with the pcDNA-ANRIL group, expression of FLT-1 was evaluated in the pcDNA-ANRIL + PDTC group). Notes: IHC, immunochemistry; FLT-1, FMS-like tyrosine kinase-1; VEGF, vascular endothelial growth factor; The Vector group, injected with 800 ng/kg empty plasmid; The shANRIL group, injected with 800 ng/kg lncRNA ANRIL knockout plasmid; The PDTC group, injected with 800 ng/kg NF-κB inhibitor pyrrolidine dithiocarbamate (PDTC); The pcDNA-ANRIL + PDTC group, injected with PDTC after lncRNA ANRIL overexpression; DM, diabetes mellitus; CI, cerebral infarction.

### Comparisons of endothelium dependent MVD in each group

DM + CI group witnessed a large number of CD31 positive staining cells; model group and over-expressed ANRIL group saw denser endothelium-dependent vessels; knockout of lncRNA ANRIL and injection of PDTC resulted in a more remarkable decrease in endothelium-dependent vessels than Vector group, whereas over-expressed lncRNA ANRIL brought about an increase in endothelium-dependent vessels, and injection of inhibitor PDTC after lncRNA ANRIL overexpression led to an decrease in endothelium-dependent vessels than over-expressed lncRNA ANRIL (Figure 7). As was revealed in Table 3, compared to Vector group, over-expressed lncRNA ANRIL led to an apparent increase in endothelium dependent MVD (*P* < 0.05), while knocked ANRIL and PDTC treatment resulted in a more obvious decrease in endothelium dependent MVD value than Vector group (*P* < 0.05). Besides, injection of inhibitor PDTC after lncRNA ANRIL overexpression led to an decrease in endothelium dependent MVD value than over-expressed lncRNA ANRIL (*P* < 0.05).

**Figure 7:** Comparisons of endothelium dependent MVD in each group by double staining (× 400) (**A**, endothelium dependent MVD in the Vector group; **B**, endothelium dependent MVD in the pcDNA-ANRIL group; **C**, endothelium dependent MVD in the shANRIL group; **D**, endothelium dependent MVD in the PDTC group; **E**, endothelium dependent MVD in the pcDNA-ANRIL + PDTC group. Compared with the Vector group, endothelium-dependent vessels were increased in the pcDNA-ANRIL group, while endothelium-dependent vessels were decreased in the shANRIL group and the PDTC group. Compared with the pcDNA-ANRIL group, endothelium-dependent vessels were increased in the pcDNA-ANRIL group.). Notes: MVD, microvessel density; CD31, differentiation 31; PAS, para-amiuosalicylic acid; PDTC, pyrrolidinedithiocarbamic acid; The Vector group, injected with 800 ng/kg empty plasmid; The shANRIL group, injected with 800 ng/kg lncRNA ANRIL knockout plasmid; The PDTC group, injected with 800 ng/kg NF-κB inhibitor pyrrolidine dithiocarbamate (PDTC); The pcDNA-ANRIL + PDTC group, injected with PDTC after lncRNA ANRIL overexpression; DM, diabetes mellitus; CI, cerebral infarction.

**Table 3:** Differences in microvessel density (MVD) of rats’ brain tissues in each group

Group	Sample number (view)	MVD
Vector	8	5.57 ± 0.56
ShANRIL	8	2.25 ± 0.21*
PDTC	8	2.11 ± 0.19*
pcDNA-ANRIL	8	9.85 ± 1.04*
pcDNA-ANRIL+PDTC	8	4.84 ± 0.87

Notes: PDTC, pyrrolidine dithiocarbamate; MVD, microvessel density; *, compared with the Vector group, P < 0.05.

## DISCUSSION

The recurrence rate, morbidity and mortality related to DM complicated with CI are high with poor prognosis [2]. As it cannot be easily detected, it is of great importance to find a biomarker. Thus, this study was initiated to address the disease from the perspective of molecular level.

It was found out in the study that lncRNA ANRIL was involved in DM complicated with CI through NF-κB signaling pathway. LncRNA ANRIL was recognized as an oncogene that was involved in a variety of diseases; however, its inhibition was proved to suppress cell proliferation, migration and invasion [8]. Activation of NF-κB, a family of transcription factors, has been revealed to take control of multiple cellular processes in diseases including inflammation, proliferation, angiogenesis, etc. [13]. Diabetic metabolic disorder including DM leads to β-amyloid protein (Aβ) generation and activation of NF-κB signaling pathway in the hippocampus, making it possible to attenuate DM complicated with CI by inhibiting NF-κB pathway [14]. IκB phosphorylation initiates subsequent dissociation and activation of NF-κB, which further translocates to nucleus [14]. And NF-κB Interacting lncRNA (NKILA), which is upregulated by NF-κB, binds to NF-kB/IκB, and directly masks IκB phosphorylation motifs, thus exerting influencing on IκB phosphorylation and NF-κB activation which further activates NF-κB signaling pathway [15]. Previous studies have reported that high lncRNA ANRIL expression had poorer overall survival compared with low lncRNA ANRIL group in a wide range of diseases, which was in accordance with our study on DM complicated with CI [10, 16]. In addition, our result was further supported by Liu *et al*. who found in their study that lncRNA ANRIL, by directly interacting with functional domains of signaling proteins, served as a class of NF-κB modulators to suppress disease metastasis [15].

The study also revealed that lncRNA ANRIL is also associated with VEGF and MVD in subjects with DM complicated with CI, with over-expression of lncRNA ANRIL resulting in increased expressions of VEGF and MVD and knockout of lncRNA ANRIL resulting in reduced expressions of VEGF and MVD. It is also possibly through NF-κB pathway that lncRNA ANRIL has impact on VEGF and MVD expressions. Angiogenesis marks an indispensable process for maintaining disease progression in hippocampus with CI, and MVD index was proven to be a prognostic factor of angiogenesis [17]. VEGF, a mitogen for endothelial cells, is the most attractive candidate for angiogenesis and vascular hyper-permeability in DM [18]. Once over-expressed lncRNA ANRIL-mediated NF-κB transcriptional activity was released, NF-κB pathway was then activated so as to result in increased production of its target-gene product, VEGF, whereas the result was abrogated after lncRNA ANRIL knockdown or using specific NF-κB inhibitor PDTC [19]. As VEGF indicated increased expression with activated NF-κB, angiogenesis would proceed, which was in turn revealed in the increase in MVD expression [20]. Choudhuri *et al.* verified in their study the relationship between NF-κB pathway activation and downstream up-regulation of VEGF in diabetic retinopathy (DR), a microvascular complication of DM, which was in accordance with our findings [21]. And the result was also supported by Polyakova who found that NF-κB inhibition resulted in functional deterioration that was associated with decreased MVD [22]. Furthermore, it was found out that knockout of lncRNA ANRIL combined with PDTC administration resulted in no change in FLK-1 expression but a decrease in FLT-1 expression. The FLK-1, a ligand of VEGF, is only limited to endothelial cells and their embryonic precursors in receptor expression, which may probably account for its stable expression in the study [23]. FLT-1 is a high affinity VEGF receptor and is regarded as specific to endothelial cells, the loss of which can lead to vessel overgrowth and dysmorphogenesis [24]. As blood vessel formation demands integrated regulation of endothelial cell proliferation and branching morphogenesis, it is possibly the ability of FLT-1 isoform that transgenes to rescue the vascular development of embryonic stem cell-derived FLT-1-mutant vessels [25].

In conclusion, the study found that the overexpressed lncRNA ANRIL up-regulated VEGF and improved angiogenesis through activation of NF-κB signaling pathway in rats with DM complicated with CI, which lays a framework for clinical treatment of DM complicated with CI based on molecular level. However, we did not select large enough samples to substantiate our conclusion and it is a study conducted in animals, it has a long way to go before applying the result to human. Therefore, more studies with larger samples need to be carried out and gradually extended to human so as to verify the result and to further elucidate the mechanisms.

## MATERIALS AND METHODS

### Ethical statement

All rats were tested in strict accordance with national animal experiment requirement that were approved by animal ethics association of The First Hospital of Jilin University. The animal used in this experiment was approved by Ethic Committee of The First Hospital of Jilin University.

### Study subjects

The study selected 112 healthy adult male Wistar rats (7-week old, weighing 260 ± 20 g) of clean grade were purchased from Institute of zoology, Chinese academy of sciences (Beijing, China). They were kept in separate cages and fed with healthy diet, at temperature of 25 ± 1°C and humidity of 50%. They were randomly divided into two groups and fed under same condition.

### Model establishment

The models were built with twice medicine injection. The experimental rats were intraperitoneally injected with 100 mg/kg alloxan for two successive days. At 72 h after last injection, the fasting blood glucose values of rats were measured by glucose oxidase method (GOD). If this value reached to 16.7 mmol/L or above, diabetic rat models were constructed. After that, they were fed with high fat diet for five successive weeks, and then were intraperitoneally injected with 20% urethane and anesthetized. Then middle cerebral artery occlusion (MCAO) models were prepared with suture method. With door temperature at 24 ± 1°C, lied on their back on the operating table, rats were cut open in the middle of neck, where right common carotid artery (CCA), external carotid artery (ECA) and internal carotid artery (ICA) were separated and exposed, and the proximal end of right CCA and the root of ECA were ligatured. At the distal end of CCA, its superior wall was pricked with needle, where a 0.25 mm nylon thread was inserted into, reaching to the base of artery through ICA. When caught up with resistance, they were fixed by suture method, and incision was sutured at last. If rats revolved toward left when walking or had left acroparalysis when they revived, their embolization was successful and can be used for the study. The rest rats were failure and not used for test.

### Plasmid construction

The plasmid pcDNA™3.1 (Invitrogen, Carlsbad, California, USA) had ampicillin resistance with 5428 bp. The design and construction of recombinant plasmids, including high expression plasmid pcDNA3.1-lncRNA ANRIL and low expression plasmid pcDNA3.1-shLncRNA ANRIL, were made by Shanghai Genechem Co., Ltd (Shanghai, China).

### Grouping and treatment method

The 112 rats were randomly divided into two groups, including DM + CI group and healthy control group, with 56 rats in each group. The rat models of control group were all successful while 46 rat models of DM + CI group were successful. After neurological severity score (NSS) and triphenylte-trazolium chloride (TTC) staining of rats, six rats of each group were randomly selected, and then these rats were killed and taken out of whole brain tissue for relevant gene protein and mRNA detection. The rest 40 rats of DM + CI group were randomly subdivided into 5 groups: Vector group (injected with 800 ng/kg empty plasmid into lateral ventricle); shANRIL group (injected with 800 ng/kg lncRNA ANRIL knockout plasmid into lateral ventricle); pyrrolidine dithiocarbamate (PDTC) group (injected with 800 ng/kg NF-κB inhibitor PDTC into lateral ventricle); pcDNA-ANRIL group (injected with lncRNA ANRIL overexpression plasmid); pcDNA-ANRIL + PDTC group (injected with PDTC after lncRNA ANRIL overexpression).

### NSS

After 4 h the rats woken from surgery, they had NSS detection. The higher score they had, the more severe the animal behavior disorder was [26]. 0 score represented no defect; 1 score indicated that front right paw cannot complete unbend; 2 scores meant that resistance to be pushed to another side was significantly decreased; 3 scores indicated that rats went around in circle spontaneously and preferred walking toward another side; 4 scores meant that rats can only walk when they were stimulated; 5 scores indicated that rats had no obvious action on stimulation and level of consciousness was decreased. The score over two was as a standard of successful model.

### TTC staining

The rats of successful models were intraperitoneally injected with 20% urethane and anesthetized. And then their brains were taken out and quick-frozen for 5 min at - 20°C refrigerator, of which the frontal pole were cut off with a sharp blade. One piece of brain tissue was sliced every 3 mm, and these slices were put into 2% TTC solution in the lucifugal cup, stored at 37°C incubator for 20 min. The stained slices were soaked in 4% paraformaldehyde and immobilized for 10 h when photos would be taken. By BI-2000 Medicine Image Analysis System (MIAS) (Olympus, Japan), the homolateral CI volume was detected, and the CI volume of each brain slice can be calculated with homolateral CI volume multiplying its thickness. The total CI volume was equal to the sum volume of five brain slices. The relative CI volume = the total CI volume/the volume of contralateral brain tissues.

### Extraction of rat tissues

The rats were intraperitoneally injected with 20% urethane and anesthetized, and then were rapidly filling with 100 ml normal saline (NS) through left ventricular to wash blood vessel. Then they were slowly injected with 200 ml 1.5 % glutaraldehyde and 200 ml 4 % paraformaldehyde for 1 hour. The equivalence region of penumbra was set by position location method between groups. The cortical tissue between 7 and 13 nm from tip of olfactory bulb in right brain as well as 1/3 cortical tissue between fissura sagittalis and lateral fissure of brain, were taken off under low temperature.

### Brain tissue slices of rats

Samples were taken out by coronal plane beyond front 2 mm and back 2 mm from optic chiasma in the brain tissues of rats, and after paraffin embedding of these samples, obvious CI parts which observed by light microscope were selected for immunohistochemistry (IHC) analysis. Brain tissue slices were dehydrated and discolored by ethyl alcohol, and then immobilized by 4% paraformaldehyde. After that, they were sliced with paraffin embedding, and followed by routine Haematoxilin-Eosin (HE) staining they were sealed with gum. Light microscope was used to observe the histological characteristics of cerebral ischemic injury as well as characteristics of neerotizing neuron. These brain tissues were immobilized by 4% paraformaldehyde for 24 h and stored at 4°C. The immobilized tissues were rinsed for 2 h, followed by which they had procedures as dehydration, transparency, wax-filling and embedding. Finally, 6 μm paraffin slice with brain coronal plane were cut off at each 100 μm distance.

### IHC

Brain tissues of rats had routine paraffin embedding with 4 μm slices. The rabbit anti VEGF (1:200) and FLT-1 (1:200) were bought from Gibco Company (Grand Island, New York, USA), Biotin- goat anti-rabbit IgG and diaminobenzidine (DAB) were all bought from DAKO Company (Glostrup, Denmark). Before dewaxing of slices, these slices were stored for 60 min at door temperature. Afterwards, these slices were soaked in dimethylbenzene and then were dewaxed and hydrated by ethyl alcohol. Washing these slices, they were added with confining liquid and stored at door temperature for 20 min. After added with 50 μL first antibody, they were stored at door temperature for 1 h. And then they were added with second antibody, followed by which they were washed and treated by DAB coloration. Next, they were counter-stained by hematoxylin for 2 min. After hydrochloric acid alcohol differentiation, they had procedures as dehydration, transparency, mounting and microscopy.

### Endothelium dependent microvessel density (MVD) detection

The endothelial cell markers cluster of differentiation 31 (CD31) and para-amiuosalicylic acid (PAS) double staining was made for sample detection. At first, they were proceeded with CD31 IHC staining, and then were developed by DAB coloration till vascular endothelial cell turned to be claybank color under microscope, at same time, they were washed. Next, slices were restored by 0.5% schiff solution for 5 min, and then washed under running water for 2 min, followed by which these slices were put into schiff solution. If these slices turned to be red under microscope, nucleus was stained for 1 min by hematoxylin. The next step was washing these samples and differentiating them. After ammonia back to blue, they were dehydrated with graded ethanol. At last, dimethylbenzene were used for transparency operation and neutral gum for mounting. Under light microscope (×100), running and direction of PAS positive capillary structure ring were observed on stained slices. By selecting richest staining area, endothelium dependent microvessels of CD31 positive tube and PAS positive tube were counted under high power lens. By 10 continued counting of endothelium dependent microvessels under high power lens without repetition, the mean value of these 10 times counting was identified as endothelium dependent MVD.

### Quantitative real-time polymerase chain reaction (qRT-PCR)

The rat brain tissues after homogenate were centrifuged by 3000 rpm for 10 min, at 4°C. Then supernatant were put into 1.5 mL EP tube which were marked with serial number. RNA was extracted by PCR kit, and 2 μg RNA of each sample were extracted for cDNA synthesis. After added with 3 μL Oligo (dT) primer, diethylpyrocarbonate (DEPC) water was added till the total volume was 13 μL, After 5 min degeneration at 70°C and put on ice for 5 min, 6 μL 5 × MLV buffer solution, 2 μL dNTP, 0.5 μL RNase inhibitor and 1.5 μL MMLV reverse transcriptase was added into them, and then DEPC water was added till the total volume was 30 μL. The condition of cDNA synthesis was as follow: at 42°C for 60 min, at 95°C for 10 min, termination reaction, stored at -40°C. The expressions of ANRIL, VEGF, fms-like tyrosine kinase (FLT-1), Kinase insert domain protein receptor (FLK-1) and reference gene GAPDH were detected by qRT-PCR. Primers were designed and synthesized by Shanghai Sangon Biological Engineering Technology & Services Co., Ltd (Shanghai, China). The cDNA were added into following real-time PCR reaction system: 10 μL SYBR Green Master (Rox) (Roche, Basel, Switzerland), 1 μL each for upstream and downstream primers, 1 μL cDNA, 7 μL DEPC water, 20 μL in total. The following reagents were blended and centrifuged, and then had real-time PCR reaction. The standard procedure of PCR amplified reaction: at 95°C for 30 s (pre-denaturation); 40 circulations: at 95°C for 5 s, at 60°C for 31 s; at 95°C for 20 s; at 60°C for 60 s; at 95°Cfor 15 s; at 60°C for 20 s (solubility curve). The solubility curve 60-90°C ensured amplification was single production. By analysis of CT value, the results were compared with reference gene GAPDH by relative method. Real-time PCR instrument (Eppendorf, Hamburg, German) was used in this study. The reagents applied in reverse transcription were bought from Promega (Madison, Wisconsin, USA). The primer sequences were showed as Table 1.

### Western blotting

An 100 mg of rats brain tissues were taken out from - 80°C freezer and its slices were put into 1.5 mL Eppendorf (EP) tube, where 1 ml animal tissue protein extraction kit were added into. Four or five times homogenate were made by ultrasonic machine till tissues were completely split, stored at 4°C refrigerator for 2 h. Afterwards, they were put into refrigerated centrifuge to centrifuge for 10 min at 10000 g/min, where supernatant were put into new EP tube and protein concentration were measured by bicinchoninic acid (BCA) protein kit (Univ-bio, Shanghai, China). Fifty μg total proteins had sodium dodecyl sulfate polyacrylamide gel electrophoresis (SDS-PAGE) for 120 min at the voltage of 70 v, and then transferred to Polyvinylidene Fluoride (PVDF) membrane. Next, they were added with 5% skim milk powder and stored for 1.5 h at door temperature. After first antibody (NF-κB antibody 1:1000, inhibitor of NF-κB (IκB) antibody 1:1000, VEGF antibody 1:1000 and glyceraldehyde phosphate dehydrogenase (GAPDH) antibody 1:2000) (Abcam, Cambridge, Massachusetts, USA) were added into them, they were incubated at door temperature for 2 h, and stored overnight at 4°C. The membrane was washed 3 times by Tris Buffered Saline with Tween (TBST). After added with horseradish peroxidase labeled rabbit anti-rat IgG (1:2500), they were incubated for 1.5 h at door temperature. After scanning imaging, protein band was analyzed with gray gel scan by Image software. The parallel test was repeated for three times.

### hematoxylin-eosin (HE) staining

The paraffin-embedded tissues were continuing sliced, followed by which they were stained with HE respectively. After HE staining of slices, pathologic changes of these tissues were observed under light microscope. The staining procedures including dewaxing, dehydration by graded ethanol for 10 min each gradient concentration, 2 times washing by double distilled water, 1 min hematoxylin staining, 3 times washing by double distilled water, differentiation and turned color back to blue, 1 min soaking in 70 %∼80 % ethyl alcohol and final 1 min eosin counterstaining. At last, expressions of angiogenesis and relevant gene were analyzed.

### Statistical analysis

Data were analyzed by SPSS19.0 statistical software (SPSS Inc., Chicago, Illinois, USA), where measurement data were represented by mean ± standard deviation (SD) (x ± s). Comparison was tested by *t* test and comparisons among groups were analyzed by one-way analysis of variance (ANOVA). If *P* < 0.05, it was considered to be statistically significant.

## References

[1] Konya H., Miuchi M., Satani K., Matsutani S., Tsunoda T., Yano Y., Katsuno T., Hamaguchi T., Miyagawa J., Namba. M. (2014). Hepatocyte growth factor, a biomarker of macroangiopathy in diabetes mellitus. World J Diabetes.

[2] Zhao L., Hu. F.X. (2014). alpha-Lipoic acid treatment of aged type 2 diabetes mellitus complicated with acute cerebral infarction. Eur Rev Med Pharmacol Sci.

[3] Guven A., Hancili S., Karatoprak E.Y., Tasel. B. (2014). Symptomatic cerebral infarction in a child with severe diabetic ketoacidosis. J Pediatr Endocrinol Metab.

[4] Katakami N., Takahara M., Kaneto H., Shimizu I., Ohno K., Ishibashi F., Osonoi T., Kashiwagi A., Kawamori R., Shimomura I., Matsuhisa M., Yamasaki. Y. (2010). Accumulation of gene polymorphisms related to plaque disruption and thrombosis is associated with cerebral infarction in subjects with type 2 diabetes. Diabetes Care.

[5] Lee H.S., Hwang. J.S. (2011). Cerebral infarction associated with transient visual loss in child with diabetic ketoacidosis. Diabet Med.

[6] Katsura K., Suda S., Abe A., Kanamaru T., Toda Y., Katayama. Y. (2012). Brain protection therapy in acute cerebral infarction. J Nippon Med Sch.

[7] Jiang Z., Sun J., Liang Q., Cai Y., Li S., Huang Y., Wang Y., Luo. G. (2011). A metabonomic approach applied to predict patients with cerebral infarction. Talanta.

[8] Li Z., Yu X., Shen. J. (2016). ANRIL: a pivotal tumor suppressor long non-coding RNA in human cancers. Tumour Biol.

[9] Wan G., Mathur R., Hu X., Liu Y., Zhang X., Peng G., Lu. X. (2013). Long non-coding RNA ANRIL (CDKN2B-AS) is induced by the ATM-E2F1 signaling pathway. Cell Signal.

[10] Hua L., Wang C.Y., Yao K.H., Chen J.T., Zhang J.J., Ma. W.L. (2015). High expression of long non-coding RNA ANRIL is associated with poor prognosis in hepatocellular carcinoma. Int J Clin Exp Pathol.

[11] Zhou X., Han X., Wittfeldt A., Sun J., Liu C., Wang X., Gan L.M., Cao H., Liang. Z. (2016). Long non-coding RNA ANRIL regulates inflammatory responses as a novel component of NF-kappaB pathway. RNA Biol.

[12] Congrains A., Kamide K., Ohishi M., Rakugi. H. (2013). ANRIL: molecular mechanisms and implications in human health. Int J Mol Sci.

[13] Chaturvedi M.M, Sung B, Yadav V.R, Kannappan R, Aggarwal B.B (2011). NF-kappaB addiction and its role in cancer: ‘one size does not fit all’. Oncogene.

[14] Cai Z, Zhao Y, Yao S, Bin Zhao B (2011). Increases in beta-amyloid protein in the hippocampus caused by diabetic metabolic disorder are blocked by minocycline through inhibition of NF-kappaB pathway activation. Pharmacol Rep.

[15] Liu B, Sun L, Liu Q, Gong C, Yao Y, Lv X, Lin L, Yao H, Su F, Li D, Zeng M, Song E (2015). A cytoplasmic NF-kappaB interacting long noncoding RNA blocks IkappaB phosphorylation and suppresses breast cancer metastasis. Cancer Cell.

[16] Lin L, Gu Z.T, Chen W.H, Cao K.J (2015). Increased expression of the long non-coding RNA ANRIL promotes lung cancer cell metastasis and correlates with poor prognosis. Diagn Pathol.

[17] Erbersdobler A, Isbarn H, Dix K, Steiner I, Schlomm T, Mirlacher M, Sauter G, Haese A (2010). Prognostic value of microvessel density in prostate cancer: a tissue microarray study. World J Urol.

[18] Ozturk B.T, Bozkurt B, Kerimoglu H, Okka M, Kamis U, Gunduz K (2009). Effect of serum cytokines and VEGF levels on diabetic retinopathy and macular thickness. Mol Vis.

[19] Vlachostergios P.J, Papandreou C.N (2013). The Bmi-1/NF-kappaB/VEGF story: another hint for proteasome involvement in glioma angiogenesis?. J Cell Commun Signal.

[20] Zhu F, Liu M, Pan Y, Wang X, Chen Y (2015). [Small hairpin RNA targeting inhibition of NF-kappaB gene in endometriosis therapy of Macaca fascicularis] [Article in Chinese]. Zhonghua Fu Chan Ke Za Zhi.

[21] Choudhuri S, Chowdhury I.H, Das S, Dutta D, Saha A, Sarkar R, Mandal L.K, Mukherjee S, Bhattacharya B (2015). Role of NF-kappaB activation and VEGF gene polymorphisms in VEGF up regulation in non-proliferative and proliferative diabetic retinopathy. Mol Cell Biochem.

[22] Javan H, Szucsik A.M, Li L, Schaaf C.L, Salama M.E, Selzman C.H (2015). Cardiomyocyte p65 nuclear factor-kappaB is necessary for compensatory adaptation to pressure overload. Circ Heart Fail.

[23] Xie L, Mao X, Jin K, Greenberg D.A (2013). Vascular endothelial growth factor-B expression in postischemic rat brain. Vasc Cell.

[24] Fan F, Wey J.S, McCarty M.F, Belcheva A, Liu W, Bauer T.W, Somcio R.J, Wu Y, Hooper A, Hicklin D.J, Ellis L.M (2005). Expression and function of vascular endothelial growth factor receptor-1 on human colorectal cancer cells. Oncogene.

[25] Kappas N.C, Zeng G, Chappell J.C, Kearney J.B, Hazarika S, Kallianos K.G, Patterson C, Annex B.H, Bautch V.L (2008). The VEGF receptor Flt-1 spatially modulates Flk-1 signaling and blood vessel branching. J Cell Biol.

[26] Zausinger S, Hungerhuber E, Baethmann A, Reulen H, Schmid-Elsaesser R (2000). Neurological impairment in rats after transient middle cerebral artery occlusion: a comparative study under various treatment paradigms. Brain Res.

